The article "Comparison of Needle-Warming Moxibustion and Other Physical Therapies for Lumbar Disc Herniation: A Meta-analysis" was published in 2022. Journal: Comput Math Methods Med.

# Comparison of Needle-Warming Moxibustion and Other Physical Therapies for Lumbar Disc Herniation: A Meta-analysis

**DOI:** 10.1155/2022/2986223

**Published:** 2022-07-28

**Authors:** Juan Wang, Chongnan Liang, Fanguang Zeng, Liang Fan, Jingqing Zhuang

**Affiliations:** ^1^Department of Surgery, Haikou Hospital of Traditional Chinese Medicine, Haikou 570216, China; ^2^Nursing Department, Haikou Hospital of Traditional Chinese Medicine, Haikou 570216, China; ^3^Massage Department, Haikou Hospital of Traditional Chinese Medicine, Haikou 570216, China; ^4^Outpatient Department, Haikou Hospital of Traditional Chinese Medicine, Haikou 570216, China

## Abstract

**Background:**

Needle-warming moxibustion (NWM) demonstrates a controversial effect on lumbar disc herniation (LDH). This study is aimed at comparing the efficacy of NWM and conventional acupuncture or other physical therapies on LDH through a meta-analysis.

**Methods:**

Potentially eligible literatures were retrieved and screened from electronic databases. The subject of the literature was a comparison of NWM and conventional acupuncture or other physical therapies for LDH. The methodological quality was evaluated by the Jadad scale. The chi-square test was used for the heterogeneity test. Subgroup analysis was used to explore the source of heterogeneity. Risk ratio (RR) or mean difference (MD) with 95% confidence interval (CI) was used to describe the effect size. The publication bias was evaluated by Egger's test.

**Results:**

The effective rate of NWM in the treatment of LDH was significantly higher than that of conventional acupuncture (RR = 1.27, 95%CI [1.18, 1.36], *P* < 0.00001) and lumbar traction (RR = 1.12, 95%CI [1.06, 1.18], *P* < 0.0001) There was no significant difference in the effective rate between NWM and electric acupuncture for LDH (RR = 1.06, 95%CI [0.98, 1.14], *P* = 0.17). VAS of LDH patients treated with NWM was lower than conventional acupuncture (MD = −1.51, 95%CI [−1.70, −1.31], *P* < 0.00001) and lumbar traction (MD = −2.64, 95%CI [−2.79, −2.49], *P* < 0.00001) but statistically insignificant with electric acupuncture (MD = −0.31, 95%CI [−0.72, 0.09], *P* = 0.13). JOA scores of LDH patients treated with NWM were higher than those with conventional acupuncture (MD = 2.24, 95%CI [1.04, 3.45], *P* = 0.0003) and lumbar traction (MD = 10.76, 95%CI [10.45, 11.07], *P* < 0.00001) but statistically insignificant with electric acupuncture (MD = 0.25, 95%CI [−0.95, 1.45], *P* = 0.69). The long-term effective rate of NWM on LDH was higher than that of conventional acupuncture (MD = 3.13, 95%CI[2.12, 4.61], *P* < 0.00001). In this study, no heterogeneity (*P* > 0.10, *I*^2^ < 50%) and publication bias (*P* > 0.05) among the literature were noted.

The article "Comparison of Needle-Warming Moxibustion and Other Physical Therapies for Lumbar Disc Herniation: A Meta-analysis" was published in 2022. Journal: Comput Math Methods Med.

**Conclusion:**

The effect of NWM on LDH was superior to traction therapy and conventional acupuncture therapy, but similar to electric acupuncture for LDH. High-quality randomized controlled trials were still needed to confirm the results.

## 1. Introduction

Lumbar disc herniation (LDH) is a chronic degenerative disease of the lumbar intervertebral disc characterized by rupture of the fibrous ring and protrusion of the internal nucleus pulposus [1]. LDH causes a series of symptoms related to stimulation or compression of the adjacent nerve roots, such as pain, weakness, and numbness in the waist and legs [1, 2]. Bowel dysfunction and paralysis may even occur in severe cases [1, 2]. The incidence of lumbar disc herniation has steadily increased over years [3]. In addition to physical discomforts, LDH could also incur psychological anxiety and depression that has become a serious social health problem [4, 5].

The current treatment for LDH include both surgical and nonsurgical modalities [6–8]. In fact, LDH generally follows a benign natural course and symptoms in most patients can be improved to a certain extent after nonsurgical treatment [9]. Nonoperative treatment included drug application, lumbar traction, manual therapy, epidural injection, massage, acupuncture, moxibustion, and wearing orthopedic braces [10–12]. Both acupuncture and moxibustion have been shown to be effective methods to alleviate lumbar intervertebral disc herniation. The underlying mechanism for the therapeutic efficacy may be related to the fact that the acupuncture or temperature stimulation could induce an analgesic effect by interfering with neurotransmitter transmission and reducing inflammatory reactions through improving the microcirculation of peripheral nerve tissue [13]. Needle-warming moxibustion (NWM) is a combination of acupuncture and moxibustion that has been widely used to treat LDH [10, 12, 14].

However, the efficacy of NWM in the treatment of LDH has been controversial. Some randomized controlled trials (RCT) have confirmed the effectiveness of NWM in treating LDH. For example, Lu et al. [14] observed that NWM can effectively alleviate the pain in patients with LDH and improve lumbar function. However, some studies hold different views. The therapeutic effect of NWM on LDH is similar to that of electric acupuncture [15]. The sample size of individual randomized clinical trials is small, and the level of evidence is low. It is necessary to conduct a meta-analysis to explore the efficacy of NWM on LDH. A previous meta-analysis [16] showed that the therapeutic effect of NWM was better than that of acupuncture. However, this study was limited by small sample size and observation indicators. It had not yet provided positive evidence for the efficacy and safety of NWM in LDH. Moreover, the study was limited to the short-term efficacy and failed to compare the long-term efficacy of the two treatment methods. In recent years, new data on NWM in the treatment of LDH have emerged that provided more references for a relevant systematic evaluation. This study collected the data from RCTs in recent years for meta-analysis to further promote the rational application of NWM in LDH by evaluating its efficacy and safety.

The article "Comparison of Needle-Warming Moxibustion and Other Physical Therapies for Lumbar Disc Herniation: A Meta-analysis" was published in 2022. Journal: Comput Math Methods Med.

## 2. Materials and Methods

### 2.1. Retrieval Strategy

We searched 6 databases, including China biology medicine disc (CBMdisc), China National Knowledge Infrastructure (CNKI), the Cochrane Library, Embase, PubMed, and Web of Science from the establishment of the database to May 25, 2022. There was no restriction on the language of published literature. The search strategy was determined by the combination of search subject words and free words: (“lumbar disc herniation” OR “intervertebral disc herniation”) AND (“needle warming moxibustion” OR “warm needle” OR “warming needle moxibustion” OR “needle warming moxibustion”).

### 2.2. Inclusion and Exclusion Criteria

The inclusion criteria were as follows: (1) the subjects were patients with LDH; (2) the control group and experimental group were both included; (3) the experimental group was treated with NWM, whereas the control group was treated with acupuncture or other physical therapy; (4) the observed outcomes included at least one of the following indicators: total effective rate, visual analysis scale (VAS) and Japanese Orthopedic Association (JOA) scores; and (5) the study type was RCT. The exclusion criteria were as follows: (1) retrospective study, (2) case reports or animal experiments, (3) the subjects who received surgical intervention, (4) duplicate publications, and (5) key data which were missing and could not be supplemented.

### 2.3. Literature Screening, Data Extraction, and Methodological Evaluation

Two researchers conducted literature retrieval independently according to the retrieval strategy. After reading the title and abstract, the literatures were screened, and then the full text was read to determine whether it was eligible for inclusion. The content extracted from the eligible literature mainly included the basic characteristics, such as the year of publication, the author, the country or region, and the demographics of the research subjects, intervention measures, and outcome indicators. The methodological quality of the included RCT was evaluated by two researchers independently according to the Jadad scale that included the generation of random sequence, randomized hiding, blinding method, withdrawal, and dropouts. Disagreements with regard to data extraction and methodological assessment were settled by consultation with a third investigator.

The article "Comparison of Needle-Warming Moxibustion and Other Physical Therapies for Lumbar Disc Herniation: A Meta-analysis" was published in 2022. Journal: Comput Math Methods Med.

### 2.4. Statistical Methods

The Revman 5.3 software was used for meta-analysis. The chi-square test was used for the heterogeneity test. The random-effects model and fixed-effects model were used to calculate the combined statistics in the presence (*P* < 0.1 or *I*^2^ > 50%) or absence (*P* ≥ 0.1 and *I*^2^ ≤ 50%) of interstudy heterogeneity, respectively. Subgroup analysis was used to explore the source of heterogeneity. The categorical and measurement data were expressed by the relative risk ratio (RR) or the mean difference (MD) with 95% confidence interval (CI), respectively. Egger's test was used to evaluate publication bias. Two-way *P* < 0.05 was statistically significant.

## 3. Results

### 3.1. Basic Information of Included Documents

According to the search strategy, 1605 articles were collected. According to the screening criteria, 1590 literatures were excluded after reading the title, abstract and full text. Finally, 15 literatures were included in the study [14, 15, 17–29]. The flow chart of literature screening is shown in Figure 1. The 15 publications were all RCTs, of which 14 were published in Chinese and 1 in English. A total of 1381 LDH patients, including 749 in the NWM group and 632 patients in the control group, were included. The basic information of literature and Jadad scores are shown in Table 1.

### 3.2. Short-Term Effective Rate of NWM Treatment

A total of 15 literatures reported the short-term effective rate of NWM in the treatment of LDH. As shown in Figure 2, no interstudy heterogeneity was noted (*χ*^2^ = 6.16, *P* = 0.63, *I*^2^ = 0%). The effective rate of NWM on LDH was higher than that of conventional acupuncture (RR = 1.27, 95%CI [1.18, 1.36], *Z* = 6.63, *P* < 0.00001). Egger's test showed no publication bias (*P* > 0.05). The treatment for the control group in 4 studies was lumbar traction, and there was no heterogeneity (*χ*^2^ = 6.02, *P* = 0.11, *I*^2^ = 50%). The effective rate of NWM in the treatment of LDH was higher than that of lumbar traction (RR = 1.12, 95%CI [1.06, 1.18], *Z* = 4.08, *P* < 0.0001). Egger's test showed no publication bias (*P* > 0.05). Similarly, no heterogeneity was noted among the 3 literatures that included electric acupuncture for the control group (*χ*^2^ = 3.14, *P* = 0.21, *I*^2^ = 36%). There was no significant difference between NWM and electric acupuncture in the effective rate of LDH (RR = 1.06, 95%CI [0.98, 1.14], *Z* = 1.38, *P* = 0.17). Egger's test showed no publication bias (*P* > 0.05).

The article "Comparison of Needle-Warming Moxibustion and Other Physical Therapies for Lumbar Disc Herniation: A Meta-analysis" was published in 2022. Journal: Comput Math Methods Med.

### 3.3. Effect of NWM Treatment on the VAS Score

A total of 8 articles reported the effect of NWM on the VAS scores in LDH patients. As shown in Figure 3, the treatment method of the control group in the 4 literatures was routine acupuncture, and there was no interstudy heterogeneity (*χ*^2^ = 5.98, *P* = 0.12, *I*^2^ = 49%). VAS of LDH patients treated with NWM was significantly lower than that of conventional acupuncture (MD = −1.51, 95%CI [−1.70, −1.31], *Z* = 15.20, *P* < 0.00001). The treatment method of the control group in the 2 literatures was lumbar traction, and there was no heterogeneity among the literature (*χ*^2^ = 0.37, *P* = 0.55, *I*^2^ = 0%). VAS of LDH patients treated with NWM was lower than that of lumbar traction (MD = −2.64, 95%CI [−2.79, −2.49], *Z* = 34.68, *P* < 0.00001). The treatment method of the control group in the 3 literatures was electric acupuncture, and there was no heterogeneity (*χ*^2^ = 1.31, *P* = 0.52, *I*^2^ = 0%). There was no significant difference in VAS between LDH patients treated with NWM and electric acupuncture (MD = −0.31, 95%CI [−0.72, 0.09], *Z* = 1.50, *P* = 0.13). Egger's test showed no publication bias for all analyses (*P* > 0.05).

### 3.4. Impact of NWM Treatment on Recent JOA Scores

A total of 7 articles reported the effect of NWM on recent JOA scores in LDH patients. As shown in Figure 4, the treatment method of the control group was routine acupuncture in 3 studies, lumbar traction in 2 studies, and electric acupuncture in another 2 studies. No interstudy heterogeneity was noted for the studies involving routine acupuncture (*χ*^2^ = 3.57, *P* = 0.17, *I*^2^ = 44%), lumbar traction (*χ*^2^ = 1.43, *P* = 0.23, *I*^2^ = 30%), and electric acupuncture (*χ*^2^ = 0.66, *P* = 0.42, *I*^2^ = 0%). JOA score of LDH patients treated with NWM was higher than that of conventional acupuncture (MD = 2.24, 95%CI [1.04, 3.45], *Z* = 3.65, *P* = 0.0003) and lumbar traction (MD = 10.76, 95%CI [10.45, 11.07], *Z* = 68.35, *P* < 0.00001) but statistically insignificant with electric acupuncture (MD = 0.25, 95%CI [−0.95, 1.45], *Z* = 0.41, *P* = 0.69). Egger's test all showed no publication biases (*P* > 0.05).

### 3.5. Comparison of Long-Term Effective Rate between NWM and Conventional Acupuncture

The patients were followed up in 6 literatures, and the long-term effective rate was obtained. There was no heterogeneity among the studies (*χ*^2^ = 5.45, *P* = 0.36, *I*^2^ = 8%). The long-term effective rate of NWM for LDH was higher than that of conventional acupuncture (MD = 3.13, 95%CI [2.12, 4.61], *Z* = 5.76, *P* < 0.00001), as shown in Figure 5. Egger's test showed no publication bias (*P* > 0.05).

The article "Comparison of Needle-Warming Moxibustion and Other Physical Therapies for Lumbar Disc Herniation: A Meta-analysis" was published in 2022. Journal: Comput Math Methods Med.

## 4. Discussion

LDH is a common and frequently encountered condition in the clinic. With the acceleration of global aging process and the rapid lifestyle, the incidence of LDH is gradually increasing. It has become a global health problem that cannot be ignored. NWM can relieve the inflammatory reaction by acupuncture combined with thermal stimulation.

We summarized the data from 15 literatures, including a total of 1381 patients with 749 treated with NWM and 632 with other physical therapy. The meta-analysis results showed that NWM was superior to conventional therapy and traction therapy in terms of the effective rate, VAS score, and JOA score. However, the therapeutic effects of NWM and electric acupuncture are similar. NWM and conventional acupuncture still have advantages in terms of long-term effective rate.

In addition to improving the treatment efficacy and relieving pain, some studies have also confirmed the efficacy of NWM in reducing inflammatory factors and improving lumbar function. Lu et al. [14] showed that serum levels of interleukin-6 and tumour necrosis factor *α* in LDH patients treated with NWM were significantly lower than those treated with routine acupuncture. The Oswestry disability index of the NWM treatment group was lower than that of the conventional acupuncture treatment group. NWM might alleviate patients' pain by reducing the level of inflammatory factors. Zai et al. [28] confirmed by enzyme-linked immunosorbent assay that the serum level of *β*-endorphin in LDH patients treated with NWM was significantly lower than that in the conventional acupuncture group. They also confirmed that NWM had shown a therapeutic advantage in the early stages of treatment. With additional course of treatment, the therapeutic effect of NWM became more significant than that of conventional acupuncture. NWM and conventional acupuncture treatment did not cause adverse events. Zheng [29] showed that compared with lumbar traction, NWM treatment could reduce the Oswestry disability index in patients with LDH. Wu [27] demonstrated that NWM treatment could reduce the level of inflammatory factors, including interleukin-6 and tumour necrosis factor- *α*, as compared with traction treatment. NWM treatment is also advantageous in improving patients' quality of life. Lin [23] confirmed that compared with conventional acupuncture treatment, NWM treatment could reduce length of hospitalizations and improve the activity of the lumbar spine. Liu [24] noted that NWM could reduce serum interleukin-6 and the level of peripheral blood neutrophils as compared with conventional acupuncture treatment.

The article "Comparison of Needle-Warming Moxibustion and Other Physical Therapies for Lumbar Disc Herniation: A Meta-analysis" was published in 2022. Journal: Comput Math Methods Med.

There was no significant difference between NWM and electric acupuncture with regard to treatment efficiency, VAS, and JOA scores in our study. The therapeutic effects of NWM and electric acupuncture on LDH were similar. Song et al. [26] considered that after the first treatment, the VAS of the NWM group was lower than that of the electric acupuncture group. However, there was no significant difference regarding the VAS score after long-term treatment between the NWM and electric acupuncture groups. After one course of treatment, there was no significant difference in VAS, JOA and effective rate between the 2 groups. Song et al. [26] found that the NWM and the electric acupuncture groups were similar in terms of disease recurrence after 1 month follow-up. Nonetheless, the NWM group often presented with an immediate effect and favorable short-term effect. Wang [15] compared the efficacy of conventional acupuncture, electric acupuncture, and NWM on LDH. The three acupuncture methods could reduce the pain of LDH patients and improve lumbar function. The therapeutic effect of NWM was similar to that of electric acupuncture, both of which were superior to that of conventional acupuncture. Shen [25] pointed out that the effective rate of electric acupuncture on LDH was lower than that of NWM. However, electric acupuncture and NWM have similar effects on pain relief.

This study suffers from several limitations. First, the quality of the included literature is low, which may have a certain impact on the results. Second, in terms of long-term efficacy, the effective rate of NWM is higher than that of conventional acupuncture. Due to the limitation of included literature, we cannot compare the efficacy of NWM, traction therapy, and electric acupuncture. Third, the observation indicators in our study are not comprehensive. More indicators, such as Oswestry disability index, straight leg elevation test, and serum inflammatory cytokine levels, are entailed to evaluate the efficacy. Fourth, we did not perform subgroup analysis by stratifying patients into subgroups according to patient age and sex, thus omitting important and clinically relevant conclusions.

In conclusion, the therapeutic effect of NWM on LDH is superior to traction therapy and conventional acupuncture. However, the efficacy of NWM is similar to electric acupuncture for LDH. High-quality RCTs are still needed to confirm the conclusion.

## Figures and Tables

**Figure 1:** Document screening flow chart.

**Figure 2:** Comparison of short-term effective rate between NWM group and control group. NWM: needle-warming moxibustion; EA: electric acupuncture.

The article "Comparison of Needle-Warming Moxibustion and Other Physical Therapies for Lumbar Disc Herniation: A Meta-analysis" was published in 2022. Journal: Comput Math Methods Med.

**Figure 3:** Comparison of recent vas between NWM group and control group. NWM: needle warming moxibustion; EA: electric acupuncture.

**Figure 4:** Comparison of JOA scores between NWM group and control group in recent treatment. NWM: needle warming moxibustion; EA: electric acupuncture.

**Figure 5:** Comparison of long-term effective rate between NWM and acupuncture. NWM: needle-warming moxibustion.

**Table 1:** Basic information of included literature and Jadad score.

Author	Year	Study type	Participants		Intervention		Jadad
			Treated	Control	Treated	Control	
Cao [17]	2011	RCT	32	30	NWM	Acupuncture	4
Chen [18]	2017	RCT	35	35	NWM	Acupuncture	6
Duo and Ba [19]	2016	RCT	140	140	NWM	Traction	5
Gao and Liu [20]	2013	RCT	78	70	NWM	Traction	6
He et al. [21]	2007	RCT	39	39	NWM	Acupuncture	6
Huang and Xie [22]	2010	RCT	48	48	NWM	Acupuncture	5
Lin [23]	2020	RCT	40	40	NWM	Acupuncture	4
Liu [24]	2020	RCT	32	32	NWM	Acupuncture	4
Lu et al. [14]	2021	RCT	50	50	NWM	Acupuncture	5
Shen [25]	2019	RCT	38	38	NWM	EA	5
Song et al. [26]	2016	RCT	60	60	NWM	EA	4
Wang [15]	2013	RCT	46	91	NWM	Acupuncture, EA	4
Wu [27]	2020	RCT	43	43	NWM	Traction	5
Zai et al. [28]	2018	RCT	30	30	NWM	Acupuncture	6
Zheng [29]	2018	RCT	45	45	NWM	Traction	4

NWM: needle warming moxibustion; EA: electric acupuncture; RCT: randomized controlled trial.

## Data Availability

The data used to support the findings of this study are available from the corresponding author upon request.
